# Cell cycle checkpoint in cancer: a therapeutically targetable double-edged sword

**DOI:** 10.1186/s13046-016-0433-9

**Published:** 2016-09-27

**Authors:** Roberta Visconti, Rosa Della Monica, Domenico Grieco

**Affiliations:** 1 IEOS, CNR, Via S. Pansini 5, 80131 Naples, Italy; 2 DMMBM, University of Naples “Federico II”, Via S. Pansini 5, 80131 Naples, Italy; 3 CEINGE Biotecnologie Avanzate, Via G. Salvatore 486, 80145 Naples, Italy

**Keywords:** Cell cycle checkpoint, Cancer drug, DNA damage, Mitosis, Chk1, Wee1, Spindle assembly checkpoint, Taxane, Vinca alkaloids, Fcp1

## Abstract

Major currently used anticancer therapeutics either directly damage DNA or target and upset basic cell division mechanisms like DNA replication and chromosome segregation. These insults elicit activation of cell cycle checkpoints, safeguard mechanisms that cells implement to correctly complete cell cycle phases, repair damage or eventually commit suicide in case damage is unrepairable. Although cancer cells appear to be advantageously defective in some aspects of checkpoint physiology, recent acquisitions on the biochemical mechanisms of the various checkpoints are offering new therapeutic approaches against cancer. Indeed, chemical manipulation of these mechanisms is providing new therapeutic strategies and tools to increase the killing efficacy of major cancer therapeutics as well as to directly promote cancer cell death. In this review we summarize developing concepts on how targeting cell cycle checkpoints may provide substantial improvement to cancer therapy.

## Background

The mechanisms of cell division and the genome itself are routinely endangered by endogenous and exogenous insults. For instance reactive oxygen species, produced during metabolic reactions, inflammation or exciting and ionizing radiations, can damage chromosomes and upset chromosome replication and segregation [1, 2]. To avoid transmission of altered genome to daughter cells, elaborate checkpoint pathways have evolved to arrest cell cycle progression and promote repair or, in case of unrepairable damage, stimulate cell death. Cancer cells are often defective in these checkpoint mechanisms [3]. Such defects very likely contribute to neoplastic transformation and progression by coupling genetic instability with resistance to apoptotic cell death. Nevertheless, the actual information on checkpoint biochemistry and its deregulation in cancer, along with the development of relative pharmacologic tools, is now offering new opportunities for cancer treatment. Here we will review how recent efforts to identify new strategies and drugs targeting cell cycle checkpoints will likely translate soon into benefit to clinical practice in oncology. As outlined in Table 1, we will focus our attention on drugs targeting key players of the S and G2/M checkpoints activated in response to DNA damage and on drugs targeting the mitotic spindle assembly checkpoint (SAC). For more details on other regulators of the DNA damage response, including microRNAs and long-non coding RNAs, and on their small molecule inhibitors the readers may refer to other publications [4–8].

**Table 1:** Cell cycle checkpoint targeting drugs

	Target	Drug	References
S and G2/M checkpoint targeting drugs			
	Chk1/2	UCN-01	[35, 37–40]
		ICP-1	[36]
		PF00477736	[41, 42]
		XL9844	[43]
		PD321852	[44]
		CEP3891	[45]
		AZD7762	[46]
		LY2603618	[47]
		Gö6976	[48]
		SCH900776 (MK-8776)	[49, 50, 53]
		CCT244747	[51]
	ATR	NU6027	[54]
	Wee1	MK-1775	[55–65]
Spindle assembly checkpoint targeting drugs			
	Microtubular β-tubulin	Taxanes, Vinca alkaloids	[68, 77]
	Wee1	MK-1775	[92]

### G1-S, S and G2/M checkpoints

The overall cellular response to damaged DNA, known as DNA damage response (DDR), is composed of sensor proteins that detect and signal DNA damage to downstream effectors that, in turn, arrest cell cycle progression and promote repair. In response to DNA damage, cell cycle checkpoints can be activated in G1 phase, in S phase and at the G2/M transition [9, 10]. In particular, the Ataxia Telangiectasia Mutated (ATM) kinase is activated by DNA double strand breaks (DSBs) and triggers the G1 checkpoint by phosphorylating and activating the Checkpoint Kinase 2 (Chk2) [11]. Chk2 inhibits Cdc25A, a phosphatase that removes inhibitory phosphorylation of the cyclin A/Cyclin-dependent kinase (Cdk)2 and cyclin E/Cdk2 complexes, preventing cells from proceeding into S phase [12]. Of note, the G1 checkpoint is critically dependent on p53. In addition, ATM induces phosphorylation of p53, reducing its affinity for the negative regulator, the ubiquitin ligase Mdm2, leading to p53 stabilization [13–15]. Stabilized p53 induces p21, that binds and further inhibits cyclin A/Cdk2 and cyclin E/Cdk2 complexes, DNA repair proteins and, upon protracted checkpoint activation, apoptotic cell death promoters [16–20].

When DNA damage occurs in S phase, arising from stalled replication forks, nucleotide excision/repair process or as intermediates of DSB resolution, the intra S phase checkpoint is activated to prevent further replication [21, 22]. The damage is sensed by the Ataxia Telangiectasia and Rad3-related (ATR) kinase that, by activating Checkpoint Kinase 1 (Chk1), induces Cdc25A proteosomal degradation, blocking further progression through S phase [23, 24]. ATR and Chk1 also trigger the G2/M checkpoint, which prevents cells with damaged DNA from entering mitosis. Mitosis onset requires activity of the master mitotic kinase cyclin B-dependent kinase 1 (Cdk1) [25]. Cdk1 catalytic activity is inhibited during the S and G2 phases through the phosphorylation on T14 and Y15 induced by the kinases Wee1 and Myt1 [26, 27]. These phosphorylations are removed at the G2/M transition by the Cdc25C phosphatase [26]. To prevent cells with damaged DNA from entering mitosis, ATR inhibits cyclin B/Cdk1 activation by stimulating the Cdk1 inhibitory kinase Wee1 and inhibiting Cdc25C via Chk1 [28, 29].

In response to DNA damage ATM and ATR not only stop cell cycle progression but also initiate DNA repair by phosphorylating several other substrates. If damage cannot be repaired, the cell destiny might be death or permanent growth arrest (senescence) [30, 31]. When cells with irreparable DNA damage are forced to enter into mitosis, they undergo permanent growth arrest or cell death through a so-called mitotic catastrophe mechanism. Although the mitotic catastrophe mechanistic details are still unclear, it has been recently proposed as an oncosuppressive mechanism, initiated during the M phase and requiring a prolonged mitotic arrest. Mitotic catastrophe results either in cells dying in mitosis or in cells reaching the subsequent G1 phase of the cell cycle and then dying or undergoing senescence. It is unclear whether mitotic catastrophe kills the cells by apoptosis, necrosis or autophagy; however, likely it is the result of simultaneous activation or sequential triggering of different cell death-inducing pathways [32]. These observations suggest that forced entry of DNA-damaged cells into mitosis may provide a substantial increase in therapeutic efficacy.

Damaging DNA with either chemo- or radiotherapy is the most frequently used strategy for treating human cancer; however, collateral DNA damage to normal cells, particularly in highly proliferative tissues, often limits clinical efficacy. Recently, starting from the observation that cancer cells that have defective checkpoints, often because of p53 pathway mutations, can still stop the cell cycle and avoid DNA damage-induced cell death by relying on the other checkpoint branches [33], a novel anticancer therapeutic strategy has begun to develop. This is based on combining DNA damaging drugs with drugs targeting the Chk1/2 pathways to force cancer cells to bypass the S and G2/M arrest and enter mitosis with DNA damage, leading to mitotic catastrophe [32, 34].

Many specific Chk1 inhibitors have been developed, that showed promising results in preclinical studies. UCN-01 and its analog ICP-1 have mostly shown efficacy in combination with drugs inducing replication stress such as the DNA cross-linker cisplatinum and the topoisomerase I targeting drugs, suggesting that the intra-S-phase checkpoint bypass is indeed a key step to chemotherapy sensitization [35, 36]. Phase I trials with the Chk1 inhibitor UCN-01 in combination with cisplatinum provided important proof of principle that a Chk1 inhibitor prevented cell cycle arrest caused by cisplatinum-induced DNA damage [37, 38]. Indeed, in cisplatinum-treated patients, UCN-01 infusion caused a drastic reduction of geminin, a biomarker of DNA damage-induced cell cycle arrest, as detected by immunohistochemistry in tumor biopsies [38]. However, phase II clinical trials with UCN-01 have been discontinued, mostly because of low target specificity and unfavorable pharmacokinetics [39, 40]. Many other Chk1 inhibitors have been developed and tested proving efficacy alone and in combination with other genotoxic drugs in preclinical settings [41–45]; however, the few tested in Phase I and Phase II trials have shown severe side effects and none or limited efficacy [46, 47]. Thus, many second-generation Chk1 inhibitors have recently been developed [48–51]. Preclinical studies have shown that second-generation Chk1 inhibitors are effective if used in combination with DNA-damaging drugs [48, 49]. Moreover, they are greatly effective at sensitizing cells to antimetabolites such as cytarabine or the pyrimidine antagonist gemcitabine [49, 50, 52]. These compounds, once metabolized, are incorporated into DNA, causing strand termination. Moreover, gemcitabine inhibits ribonucleotide reductase, thus depleting dNTP pool and inhibiting DNA synthesis. As Chk1 is required to stabilize the stalled replication forks, it is hypothesized that the second-generation Chk1 inhibitors cause replication fork collapse and DNA double strand breaks. Recently the phase I clinical trial results of the second generation Chk1 inhibitor SCH900776 in association with antimetabolite drugs have been reported showing promising, preliminary evidence of clinical activity in small groups of patients [50, 53]. SCH900776 is currently undergoing testing in a phase II trial in association with cytarabine in adult leukemia patients.

To target the S and G2/M checkpoint, a potent, selective ATR inhibitor, NU6027, has been developed and preclinical studies in breast and ovarian carcinoma cell lines show promising results. NU6027, in fact, was not cytotoxic as single agent; however, the drug acted to sensitize tumor cells to a variety of genotoxic insults, including ionizing radiation, cisplatinum and doxorubicin, among others [54].

Wee1 is a crucial kinase that prevents the onset of mitosis in cells that have incompletely replicated or have damaged genomes. In case of DNA damage, ATR-activated Wee1 arrests the cells at the G2/M checkpoint, allowing time for repair [28]. A Wee1 small-molecule inhibitor, MK-1775, a pyraxolo-pyrimidine derivative, is already available for oral administration and several preclinical studies have demonstrated its potency and selectivity for Wee1 (with an IC_50_ of 5 nmol/L) [55]. MK-1775, by abrogating the G2/M checkpoint, allows cells with damaged DNA to progress into mitosis, leading to mitotic catastrophe. Thus, most of the preclinical studies have tested MK-1775 in combination with DNA damaging drugs. Indeed, MK-1775 has been shown to synergize with a wide variety of DNA damaging agents (such as radiation [56], the topoisomerase inhibitor doxorubicin [57], the anti-metabolite 5-fluorouracil [57], the DNA cross-linker cisplatinum [55]). As expected, MK-1775 cytotoxicity was more pronounced in p53 minus, G1 checkpoint-deficient cells that are strictly dependent on the G2/M checkpoint to avoid mitotic entry with DNA damage and, in turn, death [55–57]. Xenograft studies in nude mice bearing cervical, ovarian, colorectal, lung, glial and pancreatic cancers have demonstrated that oral administration of MK-1775 in combination with several DNA damaging agents induces tumor regression [55, 56, 58, 59]. Phase I trials testing MK-1775 in combination with DNA damaging drugs have shown promising results, as the toxicity was easily manageable. Currently several phase II trials are underway [60].

Besides its key role in the G2/M checkpoint, Wee1 kinase controls proper timing of mitosis onset by performing inhibitory phosphorylation of Cdk1 [26]. Accordingly, using sarcoma cell lines and patient-derived tumor explants, it has been demonstrated that MK-1775, by inducing premature mitosis entry, has cytotoxic effects even when utilized as single agent [61]. On the basis of the Wee1 role in mitosis entry regulation, a novel therapeutic regimen has been suggested by combining MK-1775 with gemcitabine that, as discussed before, by targeting ribonucleotide reductase, depletes dNTP pool, thus inhibiting DNA synthesis. MK-1775 forced gemcitabine-arrested cells into mitosis without completing S-phase thereby resulting in extensive DNA damage, micronuclei formation and ultimately apoptotic death [62].

Of note, it has been demonstrated that Wee1 also regulates initiation and progression of DNA replication forks, preventing DNA double strand breaks during replication [63]. Thus, it has been suggested that MK-1775 might kill the cells by inducing DNA double stand breaks as a consequence of deregulated DNA replication rather than premature mitosis [64]. Accordingly, MK-1775 cytotoxicity does not correlate with the mitotic indexes of several cancer cell lines [64].

Irrespective of the controversial mechanism, a phase I single agent study of MK-1775 in patients with advanced solid tumors has been carried out to assess safety, tolerability and pharmacokinetics of the drug [65]. The only reported dose-limiting toxicities were supraventricular tachyarrhythmia and myelosuppression. Of twenty-five enrolled patients, two carrying BRCA mutations (one with head and neck cancer and one with ovarian cancer) showed partial responses. The trial has also evaluated the MK-1775 effects on pY15-Cdk1 (reduction in two of five paired tumor tissue biopsies) and on DNA damage markers (increase in γH2AX levels in three of five tumor tissue paired biopsies). The results indicated that MK-1775 induced stalled replication forks and DNA double strand breaks.

### The spindle assembly checkpoint

In mitosis, correct partitioning of replicated genome is granted by a safeguard mechanism, called Spindle Assembly Checkpoint (SAC), that prevents errors in chromosome segregation by delaying progression into anaphase until mitotic spindle assembly completion. SAC inhibits the ubiquitin ligase anaphase-promoting complex/cyclosome (APC/C) and delays degradation of cyclin B and of the anaphase inhibitor securin until bipolar attachment of all chromosome pairs [66]. SAC is imposed by the recruitment to unattached or tensionless kinetochores (the proteinaceous centromeric structures that interact with spindle microtubules) of the Mitotic Checkpoint Complex (MCC). MCC is composed by the proteins BubR1, Bub3 and Mad2 associated with the essential APC/C coactivator Cdc20 [67]. SAC is activated by taxanes (Paclitaxel, Docetaxel, etc.) and vinca alkaloids (Vinblastine, Vincristine, etc.), which are among the most widely used anticancer drugs. These drugs are referred to as anti-microtubule cancer drugs (AMCDs). They bind β-tubulin and affect microtubule dynamics and mitotic spindle assembly. The taxanes stabilize pre-existing microtubules, while the vinca alkaloids prevent microtubule polymerization [68]. Thus, in their presence, malformed or incomplete spindles activate the SAC. Cells held in mitosis by AMCDs-induced SAC undergo apoptosis after prolonged mitotic duration [69]. Although Cdk1 phosphorylates and inhibits caspase 9 (thereby protecting against apoptosis during normal mitosis), caspase 9 ultimately becomes dephosphorylated upon prolonged arrest in mitosis [70]. In addition, it has been demonstrated that prolonged activity of cyclin B/Cdk1 causes degradation of the antiapoptotic protein Mcl1, leading to caspase-dependent cell death of AMCDs-treated cells [71]. Moreover, Cdk1 has a role in the inhibition of the anti-apoptotic proteins Bcl-X_L_ and Bcl-2 [72, 73]. Thus, the SAC arrest-dependent apoptosis induced by AMCDs provides a mechanistic rationale for the therapeutic use of these drugs. However, cancer cells can also slip through mitosis, despite malformed spindles, by adapting to the SAC. Slippage occurs because, despite an active SAC, cyclin B is slowly degraded to levels below that needed to sustain Cdk1 activity and the mitotic state [74]. A recently developed model suggests that proapoptotic signals accumulate during AMCDs-induced prolonged mitosis; however, cells can survive the treatment if they slip through mitosis before a certain proapoptotic signal threshold has been reached [75]. Conversely, if the threshold is reached before slippage, cells die [75, 76]. Most of the cells that slip through mitosis either stop dividing in a tetraploid G1 state, become senescent, or die at later stages [76]. Nevertheless, a small fraction of slipped cancer cells, especially if p53-negative, may continue dividing, thus, resisting the treatment and generating further aneuploidy via aberrant mitosis [75, 76]. By generating higher genomic instability rates, this process predisposes, in principle, cells to the acquisition of a more malignant phenotype (development of metastatic capability, drug resistance, etc.). Thus, mitotic slippage is believed a crucial mechanism for the development of resistance to AMCDs, in addition to the first described enhanced activity of MDR efflux pumps [69, 75–77]. AMCDs clinical benefits are curtailed not only by resistance but also by significant, dose-limiting, collateral damage [68, 78]. The most relevant side effects are neutropenia, consequence of toxicity on hematopoietic precursor cells, and peripheral neuropathy, due to the critical role of microtubules in neuronal axoplasmic transport [68]. To circumvent side effects, in particular peripheral neuropathy, new strategies to arrest mitotic progression without directly affecting microtubule physiology have been implemented. Indeed, a new class of drugs targeting kinesin motor proteins, that are crucially required for bipolar spindle assembly, are currently under clinical trials. It is noteworthy, however, that to date the clinical trials for this novel mitosis-targeting drugs have not confirmed the promising effects seen in preclinical models as single agents [79–83]. As an additional strategy to target mitosis, a large number of molecules has been developed and evaluated to inhibit Plk1, Aurora A and Aurora B kinases as their inactivation results in gross aneuploidy, by lack of chromosome segregation, and eventual cell death [84–86]. Nevertheless, initial clinical trials with Plk and Aurora inhibitors have not confirmed the promising preclinical data [87]. Therefore, the actual improvement in cancer cell killing efficiency of several, new mitosis-targeting compounds still wait to be established [79, 87]. Thus, novel therapeutic regimens, perhaps combining AMCDs with other drugs that prevent mitotic slippage, are needed to improve cancer cell killing efficiency helping to limit resistance occurrence and reduce side effects.

### A novel combined therapy targeting SAC-induced arrest in mitosis

Besides side effects and resistance, AMCDs are still among the most successful anti-tumor drugs, validating mitotic spindle as an excellent target for cancer chemotherapy. Thus, much effort has been directed to developing novel inroads that target spindle assembly and dynamics to improve AMCDs efficacy. A novel mitosis-targeting therapeutic approach is here proposed, based on our recent findings on mechanisms regulating mitosis exit and the SAC. We recently unveiled a novel, transcription-independent, crucial role for the essential RNA polymerase II-carboxy-terminal domain phosphatase Fcp1 in bring about Cdk1 inactivation at the end of mitosis [88–90]. We identified cyclin B degradation pathway components, like Cdc20 and the deubiquitinating enzyme USP44, and the Cdk1 inhibitory kinase Wee1 as crucial Fcp1 targets. At mitosis exit, Fcp1 promoted inhibitory Cdk1 phosphorylation by dephosphorylating Wee1, and ubiquitin-dependent cyclin B degradation by dephosphorylating Cdc20 and USP44. This lead us to hypothesize that, during prolonged mitosis in AMCDs-treated cancer cells, progressive Fcp1-induced Wee1 reactivation might lead to progressive loss of Cdk1 activity that weakens the SAC to a point in which the mitotic state could not be sustained [91]. This will translate into mitotic slippage, survival and AMCDs-resistance. Indeed, we validated this hypothesis by demonstrating that, in AMCDs-treated cells, SAC slippage depends on Fcp1-Wee1-Cdk1 (FWC). In Paclitaxel- or Vincristine-treated cells, in fact, progressive Fcp1-dependent Wee1 dephosphorylation lead to Cdk1 inactivation, SAC slippage and mitotic exit [92]. Remarkably, siRNA down modulation of Fcp1 or Wee1 significantly delayed slippage and mitotic exit in AMCDs-treated cells. Moreover, the anti-apoptotic Mcl1 protein levels were reduced to a minimum and apoptotic cell death was substantially augmented. Thus, inhibiting the FWC axis can sustain the SAC-dependent mitotic delay induced by AMCDs, substantially delaying slippage and increasing AMCDs therapeutic efficacy. Wee1 is inhibitable by orally available drugs such as MK-1775; therefore our data present a rational framework for testing the therapeutic efficiency of AMCDs in combination with Wee1 inhibitors. Indeed, we have shown that MK-1775 treatment greatly enhanced mitotic arrest, Mcl1 degradation and caspase-dependent apoptosis in several Paclitaxel-treated cell lines as well as in Vincristine-treated primary lymphoblastic leukemia cells [92]. Moreover, we predict that the combination MK-1775 plus AMCDs may allow substantial reduction of AMCDs dosage. This approach may also reduce collateral damage in patients without loosing overall AMCDs therapeutic efficacy. Therefore, the observation that the FWC axis plays a critical role in SAC slippage and mitotic exit in AMCDs-treated cancer cells provides a strong rationale for the use of MK-1775 in combination with AMCDs.

## Conclusions

DNA- and mitotic spindle-damaging drugs still remain mainstream in cancer therapy. However, it has become progressively clear that cancer cells have defective cell cycle checkpoints. These defects, which very likely contribute to neoplastic transformation and progression by increasing genetic instability, can be exploited to envision strategies that will increase our armoury against cancer.

As recapitulated in Fig. 1 and extensively discussed in the review, Chk1/2, ATR or Wee1 inhibitors can sensitize cancer cells to DNA damaging drugs forcing the cells with DNA damage to bypass the S and G2/M arrest and enter mitosis, leading to cell death by mitotic catastrophe. Strong preclinical evidences for the use of checkpoint targeting drugs alone or in combination with standard radio and/or chemotherapy have been accumulating during the recent years. It has to be noticed, however, that many Phase I trials have been terminated for toxicity and/or low target specificity, or merely for business reasons. Few Phase I trials, though, do have helped in selecting the drugs well tolerated and with some preliminary clinical efficacy. Thus, now we eagerly wait for the results of the ongoing Phase II trials.

**Fig. 1:** Targeting the cell cycle checkpoints in cancer. **a** Chk1/2 or ATR inhibitors in combination with DNA damaging drugs forces cancer cells with DNA damage to bypass the S and G2/M checkpoint arrest and enter mitosis, leading to cell death. **b** Wee1 inhibitors in combination with DNA damaging drugs forces cancer cells with DNA damage to bypass the G2/M checkpoint arrest and progress into mitosis, leading to cell death. **c** Wee1 inhibitors sustain the SAC-dependent mitotic delay induced by AMCDs, substantially increasing AMCDs therapeutic efficacy

As an alternative approach to the challenging testing of new drugs alone or in combination with standard therapy, we have here proposed the combinatory use of two already clinically usable drugs, the Wee1 inhibitor MK-1775 and AMCDs, on the basis of the novel role we unveiled for Wee1 in regulating mitosis exit. Our preclinical studies have demonstrated that MK-1775 limits AMCDs resistance; moreover, we predict that MK-1775 will allow substantial dosage reduction of AMCDs, decreasing their side effects. By suggesting that Wee1 inhibitors could be beneficial in combination with AMCDs, our data may further expand our options for cancer treatment. In particular, we hypothesize that the association of Wee1 inhibitors with AMCDs could be potentially beneficial in several cases, in which AMCDs are used as monotherapeutic agents as, for instance, in second line therapeutic regimens for several hematological and solid tumors.

## Abbreviations

AMCDs: Anti-microtubule cancer drugs
APC/C: Anaphase-promoting complex/cyclosome
ATM: Ataxia telangiectasia mutated
ATR: Ataxia telangiectasia and Rad3-related
Cdk: Cyclin-dependent kinase
Chk: Checkpoint kinase
DDR: DNA damage response
DSBs: Double strand breaks
FWC: Fcp1-Wee1-Cdk1
MCC: Mitotic checkpoint complex
SAC: Spindle assembly checkpoint
